# Targeting DNA-Protein Crosslinks *via* Post-Translational Modifications

**DOI:** 10.3389/fmolb.2022.944775

**Published:** 2022-07-04

**Authors:** Xueyuan Leng, Julien P. Duxin

**Affiliations:** The Novo Nordisk Foundation Center for Protein Research, Faculty of Health and Medical Sciences, University of Copenhagen, Copenhagen, Denmark

**Keywords:** DNA-protein crosslink (DPC), post-translational modifications (PTMs), ubiquitylation, small ubiquitin-related modifier (SUMO), poly(ADP-ribosyl)ation, DNA replication, DNA repair

## Abstract

Covalent binding of proteins to DNA forms DNA-protein crosslinks (DPCs), which represent cytotoxic DNA lesions that interfere with essential processes such as DNA replication and transcription. Cells possess different enzymatic activities to counteract DPCs. These include enzymes that degrade the adducted proteins, resolve the crosslinks, or incise the DNA to remove the crosslinked proteins. An important question is how DPCs are sensed and targeted for removal *via* the most suited pathway. Recent advances have shown the inherent role of DNA replication in triggering DPC removal by proteolysis. However, DPCs are also efficiently sensed and removed in the absence of DNA replication. In either scenario, post-translational modifications (PTMs) on DPCs play essential and versatile roles in orchestrating the repair routes. In this review, we summarize the current knowledge of the mechanisms that trigger DPC removal *via* PTMs, focusing on ubiquitylation, small ubiquitin-related modifier (SUMO) conjugation (SUMOylation), and poly (ADP-ribosyl)ation (PARylation). We also briefly discuss the current knowledge gaps and emerging hypotheses in the field.

## Introduction

DNA-interacting proteins become crosslinked to DNA by endogenous or exogenous sources including reactive chemicals (e.g., aldehydes), physical agents (e.g., ultraviolet (UV) light and ionizing radiation (IR)), chemotherapeutics (e.g., topoisomerase poisons and cisplatin-based compounds), and DNA damages (e.g., abasic sites). These lesions are highly diverse in the nature and size of the crosslinked protein, the chemical properties of the covalent linkage, and the structure of the linked DNA. DPCs are commonly classified as enzymatic DPCs, for DNA acting enzymes that remain stalled as covalent intermediates during their catalytic cycles, and non-enzymatic DPCs, for proteins that become linked to DNA *via* crosslinking agents (Stingele and Jentsch, 2015).

Non-enzymatic DPCs are generated in cells by crosslinking agents such as reactive aldehydes. Formaldehyde, the byproduct of histone demethylation or lipid peroxidation, covalently links proteins to DNA through a methylene bridge (Esterbauer et al., 1982; Shi et al., 2004; Lu et al., 2010). Formaldehyde is abundant in human blood and might be the major DPC inducer in cells (Heck et al., 1985; Luo et al., 2001; Nakamura and Nakamura, 2020). Highlighting the physiological relevance of formaldehyde, recent evidence in mice suggests that formaldehyde drives the phenotype of Cockayne syndrome, a disease caused by dysfunctional transcription-coupled nucleotide excision repair (TC-NER), suggesting that TC-NER may play a central role in removing formaldehyde-induced DPCs and/or other DNA lesions (e.g., DNA intra- or inter-strand crosslinks) (Mulderrig et al., 2021). Non-enzymatic DPCs can also form between nucleophilic amino acids of proteins and the open chain conformation of native apurinic/apyrimidinic (AP) sites or with the repair intermediates of certain DNA base modifications (e.g., N7-methyl-dG, N3-methyl-dA, oxidized DNA 8-oxo-dG, or modified DNA base 5-formylcytosine) (Li et al., 2017; Bai et al., 2018; Yang et al., 2018; Yang et al., 2019). Exogenous DNA damaging agents such as UV light, IR, and chemotherapeutics such as cisplatin-based compounds, can also crosslink proteins to DNA (Chodosh, 2001; Barker et al., 2005; Chvalova et al., 2007). Despite the abundance of crosslinking agents present in cells, the biological relevance of non-enzymatic DPCs is largely undetermined. This is because the protein identities and chemical properties of non-enzymatic DPCs remain poorly defined despite recent advances in mass spectrometry techniques that can quantify and monitor these DPCs in cells (Tretyakova et al., 2015; Groehler et al., 2017; Liu et al., 2018; Tayri-Wilk et al., 2020). Moreover, these agents also generate other predominant DNA lesions (e.g., DNA breaks and DNA-DNA crosslinks), making it difficult to assess the impact of non-enzymatic DPCs on cellular sensitivity and the DNA damage response using these pleiotropic crosslinkers.

In contrast to non-enzymatic DPCs, enzymatic DPCs can be induced to generate specific lesions in cells. For example, the catalytic cycles of topoisomerase 1 and 2 (TOP1 and TOP2) can be interrupted by chemotherapeutic agents (e.g., topotecan and etoposide, respectively), stabilizing the covalent links to DNA and forming topoisomerase cleavage complexes (TOP1/2-ccs, also known as TOP1/2-DPCs) (Liu et al., 1996; Champoux, 2001). The resulting 3′- and 5′-phosphotyrosyl bonds (3′-pY and 5′-pY) that link TOP1 and TOP2 to DNA can be hydrolyzed by specialized tyrosyl-DNA phosphodiesterase 1 and 2 (TDP1 and TDP2), respectively (Yang et al., 1996; Cortes Ledesma et al., 2009). Topoisomerase DPCs can also be generated *via* self-trapping mutations (e.g., *E. coli* topoisomerase I R321K/F/L or human topoisomerase 3B R338W) that inhibit the resealing step in their catalytic cycles (Narula et al., 2011; Saha et al., 2020). Similarly, the flippase recombinase (Flp) mutant H305L site-specifically crosslinks to a FRT recognition site *via* a 3′-pY, mimicking TOP1-DPCs (Nielsen et al., 2009). In analogy to TOP2, SPO11 induces concerted DSBs to initiate meiotic recombination by forming cleavage complexes that covalently link the catalytic tyrosines to DNA through 5′-Ys (Keeney et al., 1997; Johnson et al., 2021; Prieler et al., 2021). Additionally, the Epstein-Barr virus protein EBNA1 covalently binds to the origin of replication site (*oriP*) to promote viral replication termination (Dheekollu et al., 2021). Enzymes with AP lyase activity can also become covalently trapped on DNA when acting on abasic sites, such as DNA polymerase *β* (Polβ) (DeMott et al., 2002), DNA-formamidopyrimidine glycosylase (Fpg) (Gilboa et al., 2002), and poly (ADP-ribose) polymerase 1 (PARP1) (Prasad et al., 2014; Prasad et al., 2020). Alternatively, abasic sites on ssDNA are rapidly crosslinked and protected by HMCES, which represents a beneficial DPC that prevents AP sites from detrimental processing (Mohni et al., 2019). Last, DNA methyltransferases, such as DNMT1 and M.HpaII, can be covalently trapped on DNA methylation sites with modified nucleotides 5′-aza-dC and 5′-fluro-dC (Santi et al., 1984; Chen et al., 1991; Maslov et al., 2012). Various DPC repair mechanisms have been identified by studying enzymatic DPCs because they form specific lesions that can be readily induced and monitored in cells. Moreover, enzymatic DPCs are of high clinical relevance and have been extensively exploited in cancer treatment using their inducing agents (e.g., topotecan and etoposide) (Topcu, 2001).

Cells utilize three strategies to repair DPCs: 1) targeting the protein to proteolysis; 2) resolving the crosslink bond by hydrolysis; 3) and/or removing the DNA encompassing the protein adduct by DNA excision (Stingele et al., 2017). These strategies are often selectively or coordinately used to repair DPCs (Kuhbacher and Duxin, 2020). Importantly, the crosslinked proteins undergo extensive modifications during the repair process, including ubiquitylation, SUMOylation, and PARylation. Emerging evidence indicates that these PTMs are part of the sensing response directing the DPC repair pathways. In recent years, it has become evident that DNA replication stalling at DPCs triggers PTMs on DPCs to target their removal. However, DPCs are also efficiently targeted for repair by PTMs in the absence of DNA replication. Below, we summarize the mechanisms by which DPCs are sensed and targeted for removal *via* PTMs conjugated and processed by corresponding PTM writers and readers (Table 1).

**TABLE 1:** DPC-modifying PTM writers and readers.

PTM	Enzyme	Functions/pathways	Investigated DPC substrates
**PTM Writers**			
Ubiquitylation	TRAIP	Replisome component, ubiquitylates target proteins in front of replication forks	M.HpaII-DPC (Larsen et al., 2019)
	RFWD3	Binds to the ssDNA associated protein RPA, ubiquitylates target proteins on ssDNA	M.HpaII-DPC (Gallina et al., 2021)
			Fpg-DPC (Gallina et al., 2021)
			HMCES-DPC (Gallina et al., 2021)
	TRIP12	PAR-targeted ubiquitin ligase, ubiquitylates PARP1	PARP1-trapping (Gatti et al., 2020)
	RNF4	SUMO-targeted ubiquitylation pathway	M.HpaII-DPC (Liu et al., 2021)
			DNMT1-DPC (Liu et al., 2021)
			TOP1-DPC (Sun et al., 2020)
			TOP2-DPC (Sun et al., 2020)
			PARP1-trapping (Krastev et al., 2022)
	TRIM41	Ubiquitylates TOP3B-DPC	TOP3B-DPC (Saha et al., 2020)
	Slx5-Slx8	SUMO-targeted ubiquitylation pathway	TOP1-DPC (Heideker et al., 2011; Steinacher et al., 2013; Nie et al., 2017)
			TOP2-DPC (Wei et al., 2017)
	CUL3	Scaffold protein in Cullin-RING E3 ligase complex	TOP1-DPC (Zhang et al., 2004)
	CUL4B	Scaffold protein in Cullin-RING E3 ligase complex	TOP1-DPC (Kerzendorfer et al., 2010)
	BRCA1	Contributes to transcription-dependent TOP1-DPC degradation	TOP1-DPC (Sordet et al., 2008)
	BMI1-RING1A	Ubiquitylates TOP2-DPC	TOP2-DPC (Alchanati et al., 2009)
	SCFβ-TrCP	SKP1-Cullin 1-F box protein	TOP2β-DPC (Shu et al., 2020)
SUMOylation	ZATT/ZNF451	SUMOylates TOP2-DPC and stimulates TDP2-mediated hydrolysis	TOP2-DPC (Schellenberg et al., 2017)
	PIAS4	SUMO-targeted ubiquitylation pathway	M.HpaII-DPC (Liu et al., 2021)
			DNMT1-DPC (Liu et al., 2021)
			TOP1-DPC (Sun et al., 2020)
			TOP2-DPC (Sun et al., 2020)
			PARP1-trapping (Liu et al., 2021; Krastev et al., 2022)
	Pli1	SUMO-targeted ubiquitylation pathway	TOP1-DPC (Steinacher et al., 2013)
	Nse2	SUMO-targeted ubiquitylation pathway	TOP1-DPC (Heideker et al., 2011)
PARylation	PARP1	PARP1 auto-PARylation limits PARP1 trapping, recruits PTUbLs or deubiquitylation enzymes	PARP1-trapping (Prasad et al., 2014; Steffen et al., 2016; Gatti et al., 2020; Kruger et al., 2020)
			TOP1-DPC (Sun et al., 2021)
**PTM Readers/Effectors**			
Ubiquitylation	Proteasome	DPC proteolysis	M.HpaII-DPC (Larsen et al., 2019)
			DNMT1-DPC (Liu et al., 2021)
			TOP1-DPC (Desai et al., 1997; Mao et al., 2000b; Desai et al., 2003; Zhang et al., 2004; Lin et al., 2008; Sordet et al., 2008; Kerzendorfer et al., 2010; Heideker et al., 2011; Steinacher et al., 2013; Nie et al., 2017; Sun et al., 2020; Sun et al., 2021)
			TOP2-DPC (Mao et al., 2001; Wei et al., 2017; Sun et al., 2020)
			TOP3B-DPC (Saha et al., 2020)
			Polβ-DPC (Quinones et al., 2015; Quinones et al., 2020)
			PARP1-trapping (Prasad et al., 2019; Gatti et al., 2020)
			Flp-DPC (Ma et al., 2019)
			HMCES-DPC (Mohni et al., 2019)
	SPRTN^a^	DPC proteolysis	M.HpaII-DPC (Larsen et al., 2019)
			TOP1-DPC (Vaz et al., 2016; Maskey et al., 2017)
			TOP2-DPC (Lopez-Mosqueda et al., 2016; Vaz et al., 2016)
			HMCES-DPC (Semlow et al., 2022)
			Formaldehyde-induced DPCs (Lopez-Mosqueda et al., 2016; Stingele et al., 2016; Borgermann et al., 2019; Ruggiano et al., 2021)
	p97	Unfoldase activity for trapped protein	PARP1-trapping (Krastev et al., 2022)
			Eos-DPC (Kroning et al., 2022)
	Ddi1/DDI2^a^	DPC proteolysis	TOP1-DPC (Serbyn et al., 2020)
			Flp-DPC (Serbyn et al., 2020)
SUMOylation	RNF4	SUMO-targeted ubiquitylation	M.HpaII-DPC (Liu et al., 2021)
			DNMT1-DPC (Liu et al., 2021)
			TOP1-DPC (Sun et al., 2020)
			TOP2-DPC (Sun et al., 2020)
			PARP1-trapping (Krastev et al., 2022)
	Slx5-Slx8	SUMO-targeted ubiquitylation	Flp-DPC (Ma et al., 2019)
			Top1-DPC (Heideker et al., 2011; Steinacher et al., 2013; Nie et al., 2017)
			Top2-DPC (Wei et al., 2017)
	TDP2	5′-Y hydrolysis	TOP2-DPC (Schellenberg et al., 2017)
	TEX264	Recruit DPC repair factors	TOP1-DPC (Fielden et al., 2020)
	Wss1	DPC proteolysis	Top1-DPC (Stingele et al., 2014)
			Formaldehyde-induced DPC (Stingele et al., 2014)
	ACRC^a^	DPC proteolysis	TOP2-DPC (Bhargava et al., 2020; Dokshin et al., 2020)
			Formaldehyde-induced DPC (Borgermann et al., 2019)
	SPRTN^a^	DPC proteolysis	TOP1-DPC (Ruggiano et al., 2021)
			Formaldehyde-induced DPC (Ruggiano et al., 2021)
PARylation	TRIP12	PARylation-targeted ubiquitylation	PARP1-trapping (Gatti et al., 2020)
	USP7^a^	Deubiquitylating enzyme	TOP1-DPC (Sun et al., 2021)

a Putative DPC-PTM readers.

## Replication-Coupled DNA-Protein Crosslink Targeting and Proteolysis

The bulkiness of crosslinked proteins makes DPCs detrimental to normal DNA processes. Thus, proteolysis is often required to reduce the bulkiness of DPCs (Vaz et al., 2017). Ubiquitylation, with certain chain types (i.e., K48/K11), can target substrate proteins for degradation by proteolysis. Indeed, ubiquitylation has been identified on many types of DPCs, rendering them permissible to degradation by the proteasome or specialized proteases. Particularly, the process of DNA replication triggers DPC ubiquitylation by replisome- and ssDNA-associated ubiquitin ligases.

### Replication-Coupled DNA-Protein Crosslink Ubiquitylation by TRAIP

Unrepaired DPCs block DNA transaction processes including DNA replication (Kuo et al., 2007; Duxin et al., 2014). Replication-coupled DPC proteolysis was first identified in *Xenopus* egg extracts using a methyltransferase-based DPC (M.HpaII) site-specifically linked to duplex DNA (Duxin et al., 2014). This finding coincided with the discovery in yeast of the first DPC protease, Wss1 (Stingele et al., 2014). In egg extracts, it was found that DPCs stall replisome translocation, which activates a series of events that ultimately leads to the degradation of the protein adduct by the metalloproteases SPRTN (the functional homolog of Wss1 in metazoans) and/or the proteasome (Larsen et al., 2019). Upon replisome-DPC collision, the DPC is first ubiquitylated by the replisome-associated ubiquitin ligase TRAIP, which stimulates the bypass of the protein adduct by the CMG helicase and the subsequent degradation of the DPC by the proteasome (Larsen et al., 2019) (Figure 1A). In the absence of TRAIP, DPC ubiquitylation is delayed but still occurs, suggesting that additional ubiquitin ligase(s) act on the DPC downstream of TRAIP (likely RFWD3; reviewed below and Figure 1B). Importantly, the function of TRAIP is not exclusive to DPC repair. TRAIP also ubiquitylates opposing CMGs that converge on DNA inter-strand crosslinks (ICLs) to stimulate ICL unhooking by the DNA glycosylase NEIL3 or to promote the unloading of CMG and subsequent repair of the ICL by the Fanconi anemia pathway (Wu et al., 2019; Li et al., 2020). TRAIP also triggers CMG unloading at stalled replisomes to enable mitotic DNA synthesis (MiDAs) (Deng et al., 2019; Priego Moreno et al., 2019; Sonneville et al., 2019). Interestingly, the AlphaFold predicted structure of TRAIP suggests a “fishing pole” like conformation made of successive long alpha helices with the ubiquitin ligase RING domain located at one end of the pole (https://alphafold.ebi.ac.uk/entry/Q9BWF2). Such conformation would be well suited for TRAIP to interact with the replisome while simultaneously reaching and targeting protein roadblocks ahead of CMG, conferring TRAIP a universal function in ubiquitylating substrates that hinder replisome translocation.

**FIGURE 1:** Targeting DPCs for Removal *via* PTMs. **(A)** A schematic illustration of TRAIP-mediated ubiquitylation of DPCs that hinder CMG progression. **(B)** CMG bypass of DPCs exposes ssDNA and likely triggers RFWD3-mediated DPC ubiquitylation that further leads to proteolysis by the proteasome and SPRTN. SPRTN protease is targeted by ssDNA/dsDNA junctions. **(C)** Putative models illustrating how HMCES-DPCs on AP sites are either ubiquitylated by RFWD3 to undergo proteasomal degradation or targeted by SPRTN *via* nascent DNA strands extended to the lesion. **(D)** Ddi1/DDI2 might target DPCs with long ubiquitin chains, presumably associated with DNA replication (top illustration). FAM111A degrades DPCs during DNA replication *via* its interaction with PCNA (bottom illustration). **(E)** The SUMO-STUbL pathway targets DPCs to degradation in the absence of DNA replication and serves as a universal repair solution for various types of DPCs and DPC-like lesions. **(F)** ZATT-mediated TOP2-DPC SUMOylation facilitates the recruitment of TDP2 to hydrolyze the covalent linkages. **(G)** Role of SUMOylation in promoting the removal of TOP1/2-DPCs and formaldehyde-induced DPCs by DPC proteases. **(H)** Ubiquitylation-mediated proteasomal degradation of crosslinked TOP3B, Polβ-, and PARP1-DPCs. **(I)** PARP1 auto-PARylation limits PARP1-traping *via* TRIP12-mediated ubiquitylation and proteasomal degradation (left illustration). PARylation stimulates TDP1 recruitment to TOP1-DPCs while also preventing their proteasomal degradation by recruiting the deubiquitylating enzyme USP7 (right illustration).

### Ubiquitylation of DNA-Protein Crosslink on ssDNA by RFWD3

Once bypassed by the CMG helicase, DPCs block DNA synthesis behind replication forks exposing ssDNA. Such ssDNA is quickly coated by the ssDNA-binding replication protein A (RPA), which associates with the ubiquitin ligase RFWD3 (Elia et al., 2015; Feeney et al., 2017). In *Xenopus* egg extracts, RFWD3 stimulates ubiquitylation of DPCs on ssDNA (i.e., M.HpaII-, Fpg-, and HMCES-DPCs), which likely further promotes their proteolysis during replication (Gallina et al., 2021) (Figure 1B). However, as seen for TRAIP, RFWD3 function is not exclusive to DPC repair. In fact, RFWD3 seems to indiscriminately ubiquitylate proteins that stably associate with ssDNA such as RPA and RAD51 to promote their turnover during replication stress (Elia et al., 2015; Inano et al., 2017). RFWD3 also stimulates DNA damage bypass of a variety of DNA lesions by promoting protein recruitment to ssDNA gaps *via* PCNA ubiquitylation (Gallina et al., 2021). In short, while TRAIP senses and stimulates the bypass or removal of obstacles such as DPCs that block CMG translocation in front of the replication fork (Figure 1A), RFWD3 does so by ubiquitylating proteins on ssDNA generated behind the fork caused by lesions like DPCs that impair DNA synthesis (Figure 1B). In contrast to TRAIP, the function of RFWD3 can be uncoupled from the replisome and may operate on RPA coated DNA gaps throughout the cell cycle (Gallina et al., 2021).

Consistent with its activity in targeting proteins on ssDNA, RFWD3 may also have an important function in removing HMCES-DPCs, which rapidly form on ssDNA AP sites behind replication forks (Mohni et al., 2019; Thompson et al., 2019). HMCES-DPCs at AP sites induced by UV were shown to be ubiquitylated and further stabilized by proteasome inhibition in cells (Mohni et al., 2019). Consistently, HMCES-DPCs on ssDNA are ubiquitylated by RFWD3 in the absence of SPRTN in *Xenopus* egg extracts (Gallina et al., 2021). Whether RFWD3 also ubiquitylates HMCES-DPCs in mammalian cells remains to be investigated. Nevertheless, it is tempting to speculate that, once crosslinked to ssDNA, HMCES-DPCs are either rapidly degraded by SPRTN (i.e., *via* nascent DNA strand synthesized up to the lesion; see below) (Semlow et al., 2022) or ubiquitylated by RFWD3 to promote their degradation (Figure 1C). However, the impacts of HMCES-DPC formation and subsequent degradation on the DNA damage tolerance response remain vastly unknown.

### Ubiquitin and Replication-Coupled DNA-Protein Crosslink Proteolysis

DPC ubiquitylation triggered by replication is essential to recruit the proteasome for DPC degradation (Figure 1B) (Larsen et al., 2019). This was shown in egg extracts by generating a M.HpaII-DPC substrate where all ubiquitin acceptor lysines were methylated, which shielded the DPC from ubiquitylation and degradation by the proteasome. Independently of the proteasome, SPRTN also degrades DPCs during DNA replication and is likely the preferred replication-coupled protease operating in cells (Lopez-Mosqueda et al., 2016; Stingele et al., 2016; Vaz et al., 2016; Larsen et al., 2019). SPRTN can process a broad spectrum of DPC and tightly associated DNA binding protein substrates both in cells and *in vitro* (e.g., TOP1/2-, HMCES-, M.HpaII-, and Eos-DPCs; formaldehyde induced DPCs; and non-covalently associated histones, PARP1, CHK1, and USP1) (Lopez-Mosqueda et al., 2016; Stingele et al., 2016; Maskey et al., 2017; Morocz et al., 2017; Borgermann et al., 2019; Halder et al., 2019; Larsen et al., 2019; Fielden et al., 2020; Saha et al., 2021; Coleman et al., 2022; Kroning et al., 2022; Semlow et al., 2022). In contrast to the proteasome, SPRTN-mediated DPC degradation still occurred in egg extracts without DPC ubiquitylation (on the methylated DPC substrate), albeit with slower kinetics (Larsen et al., 2019). This indicates that although DPC ubiquitylation likely stimulates SPRTN activity, it is not strictly required to target SPRTN to the DPC. Instead, SPRTN is activated by nascent DNA strands synthesized up to the lesion (Larsen et al., 2019). By binding to ssDNA and dsDNA simultaneously *via* two distinct DNA binding domains (ZBD and BR, respectively) (Reinking et al., 2020b), SPRTN activity is safely localized to ssDNA/dsDNA junctions that are generated behind the replication fork (Larsen et al., 2019; Reinking et al., 2020b) (Figure 1B). Notably, SPRTN ZBD appears to shield its metalloprotease active site when SPRTN is unbound to DNA, representing another layer of regulation that activates the protease upon DNA binding (Li et al., 2019). These mechanisms safeguard essential replisome components from promiscuous SPRTN activity and are consistent with CMG’s remarkable capacity to bypass DPCs encountered on its translocating strand (Sparks et al., 2019). Moreover, SPRTN activity also requires its UBZ domain, which suggests that ubiquitylation on proteins other than the DPC may further help SPRTN localize behind the fork (Morocz et al., 2017; Larsen et al., 2019). SPRTN can also be deactivated by degradation and autocleavage *via* a mono-ubiquitylation switch, which can be antagonized by the deubiquitylating enzymes USP7, VCPIP, and/or USP11 (Huang et al., 2020; Perry et al., 2021; Zhao et al., 2021). In summary, replisomes act as sensing machineries that detect DPCs and elicit their degradation *via* direct ubiquitylation but also by generating intermediates that activate the DNA structure-specific protease SPRTN (Figure 1B). As observed for DNA replication, DPCs also block RNA polymerases during DNA transcription (Desai et al., 2003; Sordet et al., 2008; Nakano et al., 2012; Ji et al., 2019). It is therefore conceivable that transcription may offer another efficient sensing mechanism that triggers PTM-mediated DPC removal.

### DNA-Protein Crosslink Removal by Other Proteases During DNA Replication

In addition to SPRTN and the proteasome, other proteases have recently been implicated in DPC removal during S-phase. The human trypsin-like protease FAM111A was first shown to associate with nascent chromatin *via* an interaction with PCNA (Alabert et al., 2014). More recently, it was shown to participate in the resolution of TOP1-DPCs and trapped PARP1 during DNA replication (Kojima et al., 2020). FAM111A’s PCNA-interacting protein (PIP) box and its protease activity appear essential for the removal of these lesions, suggesting that PCNA recruits FAM111A during DNA replication to process protein roadblocks that impede DNA synthesis (Kojima et al., 2020) (Figure 1D). While it is still unknown whether PTMs, such as ubiquitylation, direct FAM111A activity, dysregulation of FAM111A protease severely impacts DNA replication and transcription highlighting the critical need to fine-tune protease activity in cells (Hoffmann et al., 2020; Nie et al., 2021). In contrast, the yeast aspartic protease Ddi1 and its human homolog DDI2 specifically cleave substrates containing long ubiquitin chains, potentially acting as a backup proteolysis pathway for substrates that escape proteasomal degradation (Dirac-Svejstrup et al., 2020; Yip et al., 2020). The protease activity of yeast Ddi1 was shown to contribute to the repair of Top1- and Flp-DPCs (Serbyn et al., 2020). Additionally, the recruitment of Ddi1 to DPCs coincides with the beginning of S-phase (Serbyn et al., 2020), suggesting that Ddi1 removes ubiquitylated DPCs during DNA replication but whether this is also the case in vertebrates remains unknown (Figure 1D). Taken together, FAM111A and Ddi1 represent two novel proteases that participate in DPC repair in S-phase, but their regulation and interplay with other replication-coupled DPC repair mechanisms warrant further investigations.

## Replication-Independent DNA-Protein Crosslink Targeting by SUMOylation

While DNA replication is an efficient way to sense and remove DPCs, recent evidence has highlighted the versatile roles of SUMOylation in triggering DPC repair independently of DNA replication. SUMO-targeted DPC resolution can be achieved either by their direct proteolysis *via* SUMO-targeted ubiquitylation, or through specialized pathways that remove SUMOylated DPCs in the absence of subsequent ubiquitylation.

### The Universal SUMO-STUbL DNA-Protein Crosslink Removal Pathway

SUMOylation of proteins can target them for degradation *via* SUMO-targeted ubiquitin ligases (STUbLs) (Prudden et al., 2007). The role of the SUMO-STUbL pathway in DPC repair was first suggested in fission yeast. It was shown that Top1-DPCs are first SUMOylated by the SUMO ligases Nse2 (NSMCE2 in humans) or Pli1 (PIAS family proteins in humans) and subsequently ubiquitylated by Slx8 (RNF4 in humans) to stimulate Top1-DPC repair in the absence of Tdp1 (Heideker et al., 2011; Steinacher et al., 2013). The same SUMO-STUbL pathway mediated by Pli1 and Slx8 was also observed on Top2-DPCs in fission yeast (Wei et al., 2017) and on Top1/2-DPCs in budding yeast, *via* Siz1 (PIAS4 in human) and Slx5-Slx8 (Sun et al., 2020). Likewise, Flp-DPCs also undergo SUMO-targeted ubiquitylation, which promotes their degradation by the proteasome (Ma et al., 2019) suggesting a conserved TOP-DPC resolution mechanism *via* the SUMO-STUbL pathway (Figure 1E). Importantly, recent advances demonstrated that this pathway also operates in human cells where SUMOylation by PIAS4 and subsequent ubiquitylation by RNF4 stimulate TOP1/2-DPC repair by proteasomal degradation (Sun et al., 2020) (Figure 1E). These findings rationalize the original observations that TOP1/2-DPCs undergo SUMO conjugation and ubiquitylation-mediated proteasomal degradation (Desai et al., 1997; Mao et al., 2000a; Mao et al., 2000b; Mao et al., 2001; Lin et al., 2008). However, whether such ubiquitin-mediated resolution of TOP-DPCs is exclusively dependent on the SUMO-STUbL pathway or whether, in some instances, SUMO-independent ubiquitin ligases act on TOP1/2-DPCs is still unclear (see below).

Recent studies in *Xenopus* egg extracts and human cells showed that the SUMO-STUbL pathway can be extended to other types of DPCs and DPC-like lesions (Figure 1E). DNA methyltransferase DPCs (e.g., DNMT1 and M.HpaII) on duplex DNA undergo extensive SUMOylation, which similarly stimulates their RNF4-mediated ubiquitylation and proteasomal degradation (Figure 1E) (Liu et al., 2021). While DPC SUMOylation in *Xenopus* egg extracts is primarily performed by PIAS4, multiple SUMO ligases appear to compensate for PIAS4 activity on DNMT1-DPCs in human cells, and this is also likely the case for TOP1/2-DPCs (Sun et al., 2020; Liu et al., 2021). Notably, DPC sensing and repair *via* the SUMO-STUbL pathway does not rely on DNA replication, underlining the autonomous function of this pathway (Liu et al., 2021). Moreover, unrepaired DPCs, due to inhibition of RNF4, evade DNA damage checkpoint signaling and cause chromosomal instability during mitosis, highlighting the need to repair DPCs that are formed post-replicatively before cell division (Liu et al., 2021). This pathway may also be critical in non-dividing cells that must sense and remove DPCs independently of DNA replication. Recently, PIAS4-RNF4 mediated repair has also been reported for non-covalently trapped PARP1 (Krastev et al., 2022), a DPC-like lesion induced by PARP inhibitors that impedes DNA processes (Murai and Pommier, 2019). Interestingly, removing trapped PARP1 *via* the PIAS4-RNF4 pathway relies on the unfoldase p97 (Figure 1E) (Krastev et al., 2022). Thus, DPCs and non-covalently trapped proteins elicit the same SUMO-ubiquitylation response. While proteolysis is essential to resolve DPCs, p97 unfoldase activity might be sufficient to release non-covalently trapped proteins from chromatin. Additionally, formaldehyde treatment of cells also induces a heavy SUMOylation response on chromatin and these cells rely on RNF4 to survive (Borgermann et al., 2019; Liu et al., 2021), supporting a universal role of the SUMO-STUbL pathway in the repair of all DPCs.

Taken together, the SUMO-STUbL pathway triggers DPC removal independently of DNA replication, suggesting that other DPC sensing mechanisms are engaged. Whereas PIAS family SUMO ligases may rely on their conserved DNA-binding SAP domain (Aravind and Koonin, 2000; Sun et al., 2020) to sense DPCs on DNA, other DNA scanning mechanisms may also exist to stimulate PIAS4 recruitment or other SUMO ligases to initiate SUMO-STUbL DPC removal. Although the SUMO-STUbL pathway appears to be a universal DPC repair solution, it may not always be the preferred choice and perhaps serves as a backup mechanism for DPCs escaping or lacking specialized repair pathways (reviewed below).

### ZATT-Mediated TOP2-DNA-Protein Crosslink Resolution

Although DPCs can be targeted for proteasomal degradation by the SUMO-STUbL pathway, a more direct proteolysis-free approach has been observed on TOP2-DPCs (Schellenberg et al., 2017). Initial observations showed that covalent TOP2 crosslinking by teniposide and non-covalent TOP2 trapping by ICRF-193 trigger a swift TOP2-SUMOylation response (Mao et al., 2000a; Isik et al., 2003). Recently, it was shown that the hydrolysis of the 5′-pY bonds of TOP2-DPCs by TDP2 is facilitated by TOP2 conformational changes induced by the SUMO ligase ZATT/ZNF451 (Schellenberg et al., 2017) (Figure 1F). TOP2 SUMOylation by ZATT recruits TDP2, which binds SUMOylated TOP2 *via* its split SUMO-interacting motif (SIM) and subsequently hydrolyzes the 5′-pYs. This pathway protects TOP2 from degradation, presumably allowing TOP2 recycling and downstream repair of the adduct-free DSB by non-homologous end-joining (NHEJ) (Gomez-Herreros et al., 2013). Thus, ZATT-dependent TOP2 SUMOylation could be considered as a safe mode of TOP2-DPC repair and perhaps the preferred choice employed by cells. This is consistent with the severe sensitivity of ZATT-deficient cells to TOP2 poisons (i.e., etoposide), which contrasts to the lack of sensitivity observed in the absence of RNF4 (Schellenberg et al., 2017; Olivieri et al., 2020). However, under certain conditions or when ZATT becomes limited because of excessive TOP2-DPC generation (e.g., upon etoposide treatment), cells may also rely on the SUMO-STUbL pathway to degrade the protein adduct. Curiously, ZATT-deficient cells are even more sensitive to etoposide than TDP2-deficient cells, suggesting that ZATT possesses TDP2-independent functions in repairing TOP2-DPCs (Schellenberg et al., 2017). This could be related to a role of ZATT in recruiting the DNA translocase PICH by SUMOylating TOP2 to promote genome stability upon replication stress (Tian et al., 2021), although whether PICH localizes in the nucleus in interphase is debatable (Nielsen et al., 2015). Yet, ZATT-mediated repair appears specific to TOP2-DPCs, highlighting the relevance and abundance of endogenous TOP2-DPCs in cells (without exogenous TOP2 poisons). Whether analogous specialized pathways operate on other abundant DPCs in the absence of proteolysis remains to be discovered.

## Role of SUMO in DNA-Protein Crosslink Removal by DNA-Protein Crosslink Proteases

In addition to its role in stimulating DPC removal *via* the STUbL pathway, DPC SUMOylation has been shown to stimulate DPC removal by DPC proteases. DPC proteases emerged as an efficient way to resolve DPCs, since the discovery of the first DPC protease Wss1 in yeast (Stingele et al., 2014). Wss1 was originally characterized as a SUMO-binding isopeptidase that cleaves SUMO-conjugated protein substrates and also removes ubiquitin from ubiquitin/SUMO hybrid chains *in vitro* (Mullen et al., 2010). Wss1 was then shown to degrade proteins entrapped on DNA including camptothecin-induced Top1-DPCs (Stingele et al., 2014). Consistent with SUMO conjugation on TOP1-DPCs (Mao et al., 2000b), the DPC protease activity of Wss1 (harboring SIM domains) is largely SUMO-targeted and associated with Cdc48/p97 activity (Stingele et al., 2014; Balakirev et al., 2015) (Figure 1G). Interestingly, a more recent study in yeast showed that the SUMO ligase Siz2 (PIAS4 in humans) SUMOylates proteins in the vicinity of DPCs to stimulate Wss1 recruitment to the lesion (Serbyn et al., 2021). Proteins associated with DNMT1 are also SUMOylated in cells following DNMT1 trapping *via* 5-aza-dC treatment (Borgermann et al., 2019). Thus, it appears that the DPC-triggered SUMO response not only occurs on DPCs but also on the proteins in close interaction with DPCs, forming a SUMO hub that boosts the recruitment of SUMO-targeted repair factors (e.g., SUMO proteases or STUbLs).

In vertebrates, the metalloproteases SPRTN and ACRC (GCNA) are phylogenetically related to yeast Wss1 (Vaz et al., 2017; Reinking et al., 2020a). Notably, while SPRTN carries a ubiquitin-binding domain (UBZ), ACRC possesses SUMO-interacting motifs (SIMs). Despite the lack of SIM, the DPC protease activity of SPRTN was recently shown to interact with SUMO- and ubiquitin-conjugated non-enzymatic DPCs during DNA replication (Ruggiano et al., 2021). Additionally, SPRTN can be recruited along with p97 to SUMO-conjugated TOP1-DPCs *via* the p97 co-factor TEX264, which associates with replication fork presumably tethering SPRTN to DPCs that block ongoing DNA replication (Fielden et al., 2020) (Figure 1G). However, the stimulatory function of SUMO on SPRTN activity has yet to be confirmed *in vitro*, and could be caused by indirect effects due to the global role of SUMOylation on DNA replication (Lecona et al., 2016; Franz et al., 2021). In contrast to SPRTN, which is expressed in different cell types, ACRC (GCNA) is mainly expressed in germ cells (Carmell et al., 2016) where it was recently shown to target TOP2-DPCs during meiosis (Bhargava et al., 2020; Dokshin et al., 2020) (Figure 1G). When ectopically expressed in mammalian cells, ACRC can be recruited to DNMT1-DPC sites *via* its SIMs and participate in DMNT1-DPC resolution (Borgermann et al., 2019). However, whether ACRC is a SUMO-targeted DPC protease remains to be formally demonstrated. In germ cells, the specialized topoisomerase-like enzyme SPO11, forms DPCs similarly to TOP2-DPCs *via* 5′-pYs to direct meiotic recombination (Keeney et al., 1997; Johnson et al., 2021; Prieler et al., 2021). SPO11-DPCs are processed *via* MRN endo/exonuclease activity, which excises the DNA crosslinked to SPO11 to initiate meiotic recombination (Neale et al., 2005; Garcia et al., 2011). Although the SUMO response on SPO11-DPCs has not yet been observed, whether ACRC processes SPO11-DPCs is an interesting object for future research. Additionally, Wss1, SPRTN, and ACRC were all shown to counteract formaldehyde-induced DPCs (Stingele et al., 2014; Borgermann et al., 2019; Ruggiano et al., 2021), consistent with the potent SUMOylation response on chromatin induced by formaldehyde (Borgermann et al., 2019; Ruggiano et al., 2021) (Figure 1G). However, whether these proteases directly act on formaldehyde-induced DPCs *via* SUMO targeting is not clear.

To sum up, while the action of Wss1 in yeast is clearly linked to the SUMO system (Stingele et al., 2014; Balakirev et al., 2015), this link has not been firmly validated for vertebrate DPC proteases. Although SPRTN can process SUMO-conjugated DPCs (Fielden et al., 2020; Ruggiano et al., 2021), its recruitment to lesions does not seem to rely on SUMOylation (Borgermann et al., 2019; Ruggiano et al., 2021) and SUMO inhibition in *Xenopus* egg extracts does not affect replication-coupled DPC proteolysis (Liu et al., 2021). ACRC, albeit harboring SIMs, has yet to be shown to process SUMOylated DPCs directly. Thus, whether SPRTN and ACRC depend on SUMOylation to remove DPCs and how they interact with the SUMO-STUbL pathway await further investigation. Considering that DPC SUMOylation can trigger activities that antagonize STUbLs (Nie et al., 2017; Wei et al., 2017), we envisage that the SUMO chain growth on DPCs might act as a timer to record the dwell time of a protein crosslinked to DNA. In this scenario, the initial SUMOylation of the DPC may first facilitate DPC resolution (i.e., by SUMO-induced crosslink reversal or by DPC proteases). However, if primary processing fails or are not available, SUMO chains extension may facilitate the downstream universal SUMO-STUbL removal pathway.

## Other DNA-Protein Crosslink Ubiquitin Ligases?

DPC ubiquitylation and degradation can be effectively stimulated by DNA replication or *via* the SUMO-STUbL pathway. However, some ubiquitin-mediated DPC degradation events have so far not been linked to either pathways. For example, although TOP1/2-DPCs are subjective to STUbL mediated repair, other ubiquitin ligases have been also implicated in their degradation. CUL3 and CUL4B, the scaffold proteins of Cullin-RING E3 ligase complexes, have been shown to counteract TOP1-DPCs and render cells resistance to TOP1 poison camptothecin (Zhang et al., 2004; Kerzendorfer et al., 2010). Another ubiquitin ligase BRCA1 has been shown to contribute to the degradation of TOP1-DPCs encountered by transcription machinery (Sordet et al., 2008). Similarly, the ubiquitylation-mediated degradation of etoposide-induced TOP2-DPCs were shown to be dependent on BMI1/RING1A and SCFβ-TrCP ubiquitin E3 ligase complexes (Alchanati et al., 2009; Shu et al., 2020). However, these findings have so far not been further validated and it remains unclear whether these ubiquitin ligases directly target TOP1/2-DPCs. Other repair-oriented DPC ubiquitylation events have also been observed on the crosslinked TOP3B R338W mutant, Polβ-DPCs, and PARP1-DPCs (Figure 1H) (Quinones et al., 2015; Prasad et al., 2019; Saha et al., 2020). In the case of trapped TOP3B, ubiquitylation was shown to be dependent on the ubiquitin ligase TRIM41, which targets TOP3B for proteasomal degradation to promote resolution of the crosslink by TDP2 (Saha et al., 2020) (Figure 1H). Although Polβ-DPCs and PARP1-DPCs have been suggested to undergo ubiquitin-mediated proteasomal degradation (Quinones et al., 2015; Prasad et al., 2019; Prasad et al., 2020; Quinones et al., 2020), the ubiquitin ligases operating on these DPCs remain unknown. Possibly these results suggest the existence of additional specialized DPC repair pathways that counteract specific DPC-types.

## PARylation as an Emerging Post-Translational Modification on DNA-Protein Crosslinks

In addition to ubiquitylation and SUMOylation, PARylation, which is catalyzed by Poly (ADP-ribose) polymerases (PARPs), mainly PARP1, has also been observed on DPCs and may represent another regulatory mechanism of DPC repair (Figure 1I). The dynamic turnover of PARylation on target proteins has been tightly connected to DNA damage repair and genome maintenance (Harrision et al., 2020; Demin et al., 2021). PARP1 is the prime target of PARylation (i.e., auto-PARylation), which stimulates PARP1 release from DNA (Muthurajan et al., 2014; Steffen et al., 2016; Kruger et al., 2020). Additionally, PARylation on PARP1 recruits the PAR-targeted ubiquitin ligase (PTUbL) TRIP12 to mediate proteasomal degradation of PARP1, further limiting PARP1-trapping (Figure 1I) (Gatti et al., 2020). Importantly, PARP-mediated PARylation is activated by DNA damage (i.e., DNA nicks, gaps or breaks) but not by intact DNA (Langelier et al., 2011; Langelier et al., 2012; Rudolph et al., 2021). This suggests that the PARylation response may be excluded from DPCs on intact duplex DNA, but may influence the resolution of DPCs flanked by DNA breaks (e.g., TOP-DPCs and DPCs on ssDNA or ssDNA/dsDNA junctions such as the ones generated during replication). Consistently, PARP1 appears to play a critical role in regulating TOP1-DPC repair. While several studies initially reported that TOP1-DPCs are PARylated by PARP1 *in vitro*, the outcome of this PARylation in cells was largely unknown (Malanga and Althaus, 2004; Yung et al., 2004; Park and Cheng, 2005). A recent work showed that TOP1-PARylation exhibits an adverse effect on TOP1-DPCs compared to its effect on PARP1 trapping (Sun et al., 2021). By inhibiting poly (ADP-ribose) glycohydrolase (PARG), sustained PARylation on TOP1-DPCs was shown to recruit the deubiquitylating enzyme USP7 to remove ubiquitylation on TOP1-DPCs, thus preventing their proteasomal degradation (Sun et al., 2021) (Figure 1I). Notably, TDP1 interacts with PARP1 and PARylation of TDP1 promotes its recruitment to damage sites for TOP1-DPC resolution (Das et al., 2014), suggesting that PARP1 plays a dual function in orchestrating TOP1-DPC repair (Figure 1I). On one side, PARylation would prevent the premature proteasomal degradation of TOP1-DPC while simultaneously stimulating TDP1 recruitment to the lesion. Following TDP1 recruitment, PARG removal of PAR chains on TOP1-DPCs would allow TOP1-DPC ubiquitylation and degradation by the proteasome and subsequent hydrolysis of the covalent linkage by TDP1. Importantly, the essential role of PARylation in regulating TOP1-DPC repair is highlighted by the synergistic effect of combining PARP inhibitors and TOP1 poisons to kill cancer cells (Murai and Pommier, 2019; Chowdhuri and Das, 2021). It is possible that PARP1 is recruited to other DPCs that are flanked by DNA breaks and exhibits additional roles in regulating DPC repair, which remains largely undiscovered.

## Discussion and Perspectives

Current frontiers of research in the DPC field have unveiled the essential roles of PTMs in orchestrating DPC resolution. However, it is worth mentioning that many DPC-forming enzymes, such as topoisomerases and PARP1, are routinely post-translationally modified when associated with DNA in a non-covalent manner. Such PTMs regulate their catalytic activity or affinity to DNA and therefore can influence the level of DPC formation, making it challenging to attribute the roles of PTMs to the formation or the repair of DPCs. While the replication machinery serves as a proficient DPC sensor by directly bumping into DPCs and targeting their removal, how DPCs are recognized in the absence of replication is still under debate. Nevertheless, SUMO appears to play a central role in directing the repair of DPCs that are not sensed by DNA replication. DPC SUMOylation either initiates cost-effective repair pathways (e.g., ZATT-TDP2 for TOP2-DPCs) (Schellenberg et al., 2017) or directly engages DPC proteases (e.g., Wss1 and ACRC) (Stingele et al., 2014; Balakirev et al., 2015; Borgermann et al., 2019). On the other hand, the SUMO-STUbL proteasome pathway functions as the universal solution to ensure DPC removal (Sun et al., 2020; Liu et al., 2021; Krastev et al., 2022). Thus, it is plausible that in the absence of replication, cells recognize DPCs by their retention times on DNA recorded by SUMO chain development and accordingly employ appropriate repair mechanisms. However, additional mechanisms that initially trigger DPC SUMOylation might be engaged, for example, through certain DNA-scanning enzymes or processes like DNA transcription, or *via* specific DNA structures and topologies, which remain to be identified.
